RETRACTED

# In Silico Identification and Mechanism Exploration of Active Ingredients against Stroke from An-Gong-Niu-Huang-Wan (AGNHW) Formula

**DOI:** 10.1155/2022/5218993

**Published:** 2022-04-05

**Authors:** Lei Song, Qihui Wu, Xiaomei Fu, Wentao Wang, Zhao Dai, Yong Gu, Yue Zhuo, Shuhuan Fang, Wei Zhao, Xiaoyun Wang, Qi Wang, Jiansong Fang

**Affiliations:** ^1^Science and Technology Innovation Center, Guangzhou University of Chinese Medicine, Guangzhou 510405, China; ^2^The Second Affiliated Hospital, Guangzhou University of Chinese Medicine, Guangzhou 510404, China; ^3^Clinical Research Center, Hainan Provincial Hospital of Traditional Chinese Medicine, Guangzhou University of Chinese Medicine, Haikou 570100, China; ^4^School of Life Sciences, University of Liverpool, Liverpool L69 3BX, UK

## Abstract

An-Gong-Niu-Huang-Wan (AGNHW) is a well-known formula for treating cerebrovascular diseases, with roles including clearing away heat, detoxification, and wake-up consciousness. In recent years, AGNHW has been commonly used for the treatment of ischemic stroke, but the mechanism by which AGNHW relieves stroke has not been clearly elucidated. In the current study, we developed a multiple systems pharmacology-based framework to identify the potential antistroke ingredients in AGNHW and explore the underlying mechanisms of action (MOA) of AGNHW against stroke from a holistic perspective. Specifically, we performed a network-based method to identify the potential antistroke ingredients in AGNHW by integrating the drug-target network and stroke-associated genes. Furthermore, the oxygen-glucose deprivation/reoxygenation (OGD/R) model was used to validate the anti-inflammatory effects of the key ingredients by determining the levels of inflammatory cytokines, including interleukin (IL)-6, IL-1*β*, and tumor necrosis factor (TNF)-*α*. The antiapoptotic effects of the key ingredients were also confirmed in vitro. Integrated pathway analysis of AGNHW revealed that it might regulate three biological signaling pathways, including IL-17, TNF, and PI3K-AKT, to play a protective role in stroke. Moreover, 30 key antistroke ingredients in AGNHW were identified via network-based in silico prediction and were confirmed to have known neuroprotective effects. After drug-like property evaluation and pharmacological validation in vitro, scutellarein (SCU) and caprylic acid (CA) were selected for further antistroke investigation. Finally, systems pharmacology-based analysis of CA and SCU indicated that they might exert antistroke effects via the apoptotic signaling pathway and inflammatory response, which was further validated in an in vitro stroke model. Overall, the current study proposes an integrative systems pharmacology approach to identify antistroke ingredients and demonstrate the underlying pharmacological MOA of AGNHW in stroke, which provides an alternative strategy to investigate novel traditional Chinese medicine formulas for complex diseases.

RETRACTED

## 1. Introduction

Globally, stroke is the primary cause of death and disability and can be divided into two major categories: ischemic stroke and hemorrhagic stroke [1, 2]. Ischemic stroke accounts for 88% of stroke cases and is defined as a state in which cerebral vessels are embolized and blood perfusion to the brain is decreased, giving rise to poor oxygen and glucose supplies [3]. Currently, tissue-type plasminogen activator (tPA) is the only approved clinical therapy for acute ischemic stroke [4]. However, the rate of disability and recurrence associated with stroke remains high, placing a burden on the economy and society worldwide.

In China, the inheritance of Chinese culture for thousands of years has been accompanied by the development of traditional Chinese medicine (TCM). Stroke is managed using multiple herbs or classical prescriptions. In recent years, an increasing number of studies have focused on exploring the efficacy of An-Gong-Niu-Huang-Wan (AGNHW) [5]. AGNHW, a patented Chinese drug approved by the China National Medical Products Administration (No. Z11020076), was first recorded in the Qing Dynasty as “Differentiation of Febrile Diseases,” and is generally prescribed for patients suffering from acute and chronic cerebral diseases, including hypoxic-ischemic encephalopathy, acute hemorrhagic stroke, viral encephalitis, cerebral paralysis, and severe craniocerebral trauma hypertensive cerebral hemorrhage [6]. Indeed, Shen et al. revealed the safety of oral administration of AGNHW for the treatment of ischemic stroke for 1 week, and AGNHW has been shown to have neuroprotective effects on ischemic reinjection of brain damage in rats [7]. Current literature evidence indicated that the mechanism of *Calculus bovis* in ischemic stroke may be related to the effective protection of neurovascular units in the brain by PI3K/Akt, HIF-1*α* and VEGF pathways [8]. Moreover, *realgar* and *cinnabar* have synergistic effects with other herbal materials of AGNHW and are necessary components of AGNHW's neuroprotective effect on cerebral ischemia-reperfusion injury [9]. In addition, two antistroke ingredients might play roles in AGNHW, including baicalin and berberine [5, 10, 11]. Baicalin was reported to attenuate focal cerebral ischemic reperfusion injury via inhibiting the activation of nuclear factor *κ*B p65, which might act as a potential neuroprotective agent in stroke therapy [10]. In vivo study also demonstrated that berberine could reduce ischemic brain injury, and this effect might be via increasing the activation of Akt/GSK signaling and claudin-5 and decreasing NF-*κ*B expression [11]. Despite that several reports had emerged, the specific efficacy and mechanism of action of AGNHW against stroke have not been comprehensively and systematically evaluated.

RETRACTED

Systems pharmacology is an emerging discipline that combines in silico network-based approaches and experimental assays, with the aim to elucidate the therapeutic mechanisms of complex diseases [12, 13]. For instance, systems pharmacology-based approaches are effective for exploring the multipharmacological effects of natural products on various diseases, such as Alzheimer's disease [14, 15]. In this study, an integrated systems pharmacology-based approach was used to identify the potential antistroke ingredients in AGNHW and explore the underlying mechanism of action (MOA) of AGNHW against stroke (Figure 1**)**. To this end, we first collected stroke-associated genes and decoded specific MOAs of AGNHW for stroke via data integration analysis, including compound-target network analysis and integrated pathway analysis. We next conducted network-based in silico prediction to identify potential antistroke ingredients in AGNHW. After evaluating the potential antistroke effects using drug-like properties and experimental validation with ischemia-reperfusion injury models in vitro, scutellarein (SCU) and caprylic acid (CA) showed better neuroprotective effects, less toxicity, and preferable drug-like properties. Finally, we constructed a subnetwork of these two compounds to explore their MOAs in stroke and subsequently validated the proposed pharmacological mechanisms in an OGD/R model in vitro.

## 2. Materials and Methods

### 2.1. Collection of the Chemical Ingredients of AGNHW

An-Gong-Niu-Huang-Wan is composed of *Calculus Bovis* (Niu huang, NH), *Bubalus bubalis* (Shui niu jiao, SNJ), *Moschus moschiferus* (She xiang, SX), *Margarita* (Zhen zhu, ZZ), *Cinnabaris* (Zhu sha, ZS), *Realgar* (Xiong huang, XH), *Coptis chinensis* (Huanglian, HL), *Scutellaria baicalensis* (Huangqin, HQ), *Gardenia jasminoides* (Zhizi, ZZI), *Curcuma aromatica* (Yujin, YJ), and *Dryobalanops aromatica* (Bingpian, BP). The bioactive compounds of the eleven herbs were collected from the following five data sources: (1) Traditional Chinese Medicine Integrated Database (TCMID) [16], (2) TCM-MESH [17], (3) TM-MC [18], (4) Traditional Chinese Medicine Systems Pharmacology (TCMSP) [19], and (5) Traditional Chinese Medicine on Immuno-Oncology (TCMIO) [20]. The compound information was extracted from the PubChem database, while structures were converted to canonical SMILES and InChiKey formats using the Open Babel (version 2.3.2) [21]. After removing the duplicates, 1,128 ingredients of AGNHW were obtained (Supplementary Table 1).

RETRACTED

### 2.2. Target Identification for AGNHW

The known targets of AGNHW were derived from our previously reported dataset [22], which includes 7,314 drug-target interactions (DTIs) connecting 751 targets and 2,388 natural products. The predicted targets of natural products were acquired via the balanced substructure-drug-target network-based inference (bSDTNBI) theory [22]. The bSDTNBI theory utilizes resource-diffusion processes with substructure-drug-target networks to prioritize potential targets for both known drugs and new chemical entities (NCEs). In this project, two parameters, *α* and *β*, were imported to balance the initial resource allocation of different node types and the weighted values of different edge types. The third parameter, *γ*, was used to balance the influence of the hub nodes. Four parameters (*α* = *β* = 0.1, *γ* = –0.5, and *k* = 2) of bSDTNBI were derived from a previous study [23]. Among the above network models, bSDTNBI_KR, which was developed using different types of fingerprints, performed best with the highest values of *P* (0.049), *R* (0.752), eP (27.02), eR (27.24), and AUC (0.959). As a result, bSDTNBI_KR was utilized to predict new targets of natural products in the global network with the top 20 predicted target candidates for each natural product.

### 2.3. Integration of Stroke Disease Genes

Stroke-associated genes were collected from the following widely recognized databases: the GWAS Catalogue (https://www.ebi.ac.uk/gwas/), DisGeNET (https://www.disgenet.org/), the Human Gene Mutation Database (HGMD: http://www.hgmd.org), the Malacards database (https://www.malacards.org), and the Comparative Toxicogenomics Database (CTD: http://ctdbase.org/). For DisGeNET, we only kept the stroke genes with a DisGENET score > 0.3 and an evidence index (EI) > 0. We searched these databases with the keyword “Stroke” [MenGen ID: C0038454] and obtained 245 stroke targets as a result (Supplementary Table 2).

### 2.4. Construction of Drug-Target Network

The drug-target (D-T) networks were constructed using the Cytoscape (version 3.2.1) and Gephi (version 0.9.2). In the present D-T network, compounds or genes are conferred by nodes, while interactions are encoded by edges. The quantitative property “degree” was calculated as multiple edges linked to each node, demonstrating the significance of a given node in a network.

### 2.5. Identification of Potential Antistroke Ingredients in AGNHW

We developed a statistical network model to prioritize the antistroke indications of ingredients via the integration of drug-target network and stroke-associated genes [24]. We assumed that a compound in AGNHW would exert high potential for the treatment of stroke if its drug targets were disease genes of stroke. Fisher's exact test was used to evaluate the statistical significance of the enrichment of stroke genes in the target profiles of each compound in AGNHW [25]. The *P* values were corrected by the Benjamini–Hochberg method and a cutoff adjusted *P* value threshold (*q*) < 0.05 was set to define the significantly predicted ingredient-stroke pairs.

RETRACTED

### 2.6. Experimental Validation

#### 2.6.1. In Vitro Cell Culture and Oxygen-Glucose Deprivation/Reoxygenation (OGD/R)

Differentiated rat pheochromocytoma (PC12) cells were obtained from the Shanghai Institute of Life Sciences, Chinese Academy of Sciences. PC12 cells were cultured in Dulbecco's modified Eagle's medium (DMEM) (Gibco, USA) containing 10% fetal bovine serum (FBS) and 1% penicillin-streptomycin in a humidified incubator at 37°C with 5% CO_2_. Caprylic acid CA (T3946), chrysin (T2837), and imperatorin (T2845) were purchased from the Aladdin, China (https://www.aladdin-e.com/). Scutellarein (SCU, T3319), fisetin (T2879), gallic acid (T0877), morin (T2835), and palmatine (T5S0802) were purchased from the Bidepharmatech, China (https://www.bidepharmatech.com/). Their respective purities were > 98.5%, and all of the reagents were dissolved in dimethyl sulfoxide (DMSO) as a stock solution at 0.1 M. The OGD/R model of PC12 cells was established as previously described [26]. Specifically, PC12 cells cultured in glucose-free DMEM were incubated at 37°C and N_2_/CO_2_ (95%/5%) in a hypoxic incubator chamber (Thermo Scientific, USA). After incubation for 4 h under hypoxic conditions, PC12 cells were transferred back to normal DMEM containing 10% FBS and 4500 mg/L glucose and subsequently incubated under normal culturing conditions to recover [27]. Control cells were not treated with OGD/R.

#### 2.6.2. Cell Viability Assay

The cell viability was determined using the MTT assay. Briefly, the cells were incubated with MTT (5 mg/ml) for 4 h after treatment. Formazan, generated by living cells, was dissolved in DMSO. The optical density (OD) was read at 490 nm using a microplate reader (Bio-Rad Model550, CA).

#### 2.6.3. Terminal-Deoxynucleotidyl Transferase-Mediated UTP Nick and Labeling (TUNEL) Staining

The TUNEL assay was conducted with PC12 cells using the One-step TUNEL Apoptosis Assay Kit (Beyotime). Specifically, PC12 cells were fixed with cold 4% paraformaldehyde for 30 min, permeabilized with 0.1% Triton X-100 for 5 min, and subsequently incubated with TUNEL reagents for 1 h at 37°C in the dark. The slides were washed with PBS and counterstained with DAPI staining solution for 5 min. TUNEL-positive cells were imaged using a fluorescence microscopy.

RETRACTED

#### 2.6.4. Annexin V/PI Staining

The detection of PC12 cell apoptosis was determined by flow cytometry. Cells from each group were harvested, washed twice with PBS, and suspended in 5 mL binding buffer. Cells were stained with 5 *μ*L Annexin V-fluorescein isothiocyanate (FITC) and PI staining solution for 15 min in the dark at room temperature, and cell apoptosis was detected by flow cytometry (BD Biosciences, USA).

#### 2.6.5. Enzyme-Linked Immunosorbent Assay (ELISA)

The cell supernatant was obtained from each group and centrifuged at 12,000 × g for 10 min. After collecting the supernatant, ELISA kits (ELISA, Biological Technology, Jiangsu) were used to detect the levels of TNF-*α*, IL-1*β*, and IL-6, as described in the ELISA kit instructions. All procedures were repeated at least 3 times.

### 2.7. Statistical Analysis

Data are expressed as the mean ± SD and were analyzed using the SPSS software (version 17.0). Comparisons for more than two groups were performed using the one-way analysis of variance (ANOVA) followed by Dunnett's post hoc test. When equal variance was not assumed, the data were compared using a nonparametric test. Statistical significance was set at *P* < 0.05.

## 3. Results

### 3.1. Overlap Analysis of Herbal Ingredients and Targets in AGNHW

The most distinctive theory of traditional Chinese medicine (TCM) prescriptions is the theory of “Jun-Chen-Zuo-Shi”. In AGNHW, each medicinal material plays different roles, independently or in combination, to ensure the smooth operation of the formula [28]. To investigate how these herbs interact with each other, an overlap analysis of herbal ingredients and targets in AGNHW was performed.  Figure 2(a) shows the relationship of the 11 medicinal materials based on the number of shared ingredients. There are several common ingredients among these herbs: Yujin (YJ, Chen medicine) displays 1 compound overlap (Borneol) with Shexiang (SX, Jun medicine) and 15 compounds overlap with Bingpian (BP, Chen medicine), suggesting that “Chen” drugs not only potentiate the “Jun” drug curing the main disease but also treat the accompanying diseases or symptoms together. Borneol, as a common ingredient in YJ, SX, and BP, is reported to play a protective role in brain ischemic damage by inhibiting inflammation and suppressing apoptosis [29].  Figure 2(b) displays the overlap of herbal targets among the 11 types of medicinal materials. YJ and BP had the highest number of shared targets (*n* = 18), followed by YJ and Huangqin (HQ, *n* = 11). Moreover, HQ, HL, YJ, and ZZ (Chen medicine) are closely connected with each other, demonstrating that they share many common targets.

RETRACTED

### 3.2. Drug-Target (D-T) Network Analysis

Next, we constructed a drug-target interaction (DTI) network by extracting the known and predicted target proteins of natural products (Supplementary Table 3). The D-T network comprises 1,350 DTIs connecting 873 compounds and 477 human proteins (Figure 3). Among the 873 ingredients, the top 10 with largest target degree (*D*) are quercetin (CID5280343, *D* = 100), quercetin-7-olate (CID46906036, *D* = 100), apigenin (CID5280443, *D* = 70), apigenin-7-olate (CID25200950, *D* = 70), genistein (CID5280961, *D* = 49), chrysin (CID5281607, *D* = 46), caffeic acid (CID689043, *D* = 43), baicalein (CID5281605, *D* = 41), and gallic acid (CID370, *D* = 40), and fisetin (CID5281614, *D* = 39). Previous studies have shown that baicalein exerts a neuroprotective effect on ischemia/reperfusion injury by altering the NF-*κ*B, LOX, and AMPK/Nrf2 pathways [30]. Apigenin has also been reported to improve cognitive impairment after cerebral ischemia-reperfusion injury through multiple mechanisms [31]. Of the 477 targets, the following 10 were targeted by more than 100 compounds: LMNA, CYP3A4, MAPT, TSHR, ALDH1A1, SMN1, CYP19A1, TDP1, RAB9A, and NPC1. Previous studies have demonstrated that these targets are closely related to the occurrence and development of stroke. Indeed, a recent study found that CYP3A4 might be a protective factor for ischemic stroke, while CYP11A1 polymorphism is likely a risk factor for ischemic stroke in the Chinese Han population [32]. Overall, this D-T network contributes to uncovering the MOA of the ingredients in AGNHW against stroke.

### 3.3. Integrated Pathway Analysis of AGNHW Related to Stroke Pathogenesis

To investigate the therapeutic mechanisms of AGNHW against stroke, we conducted a pathway enrichment analysis of the overlapped targets between AGNHW and stroke using the DAVID database [33]. Detailed pathway information is provided in Supplementary Table 4. The pathways directly associated with stroke were integrated into Figure 4 based on target prediction and stroke pathology. As described in Figure 4, three typical pathways were involved in the mechanism of action of AGNHW against stroke, including the interleukin (IL)-17 signaling pathway, TNF signaling pathway, and the PI3K/AKT signaling pathway, all of which have been reported to participate in the regulation of a variety of biological processes, including cell proliferation [34], apoptosis [35], inflammation [36], and survival growth [34]. All of these pathways are closely related to the pathogenesis of stroke. For instance, the PI3K/AKT signaling pathway regulates several biological processes, and the expression of PI3K/AKT is upregulated in the central nervous system, which is beneficial to nerve cells and effectively reduces cell mortality [37, 38]. As shown in Figure 4, PTGS2, a key protein in the TNF signaling pathway, is targeted by AGNHW. Silencing of PTGS2 has been shown to inhibit apoptosis and promote proliferation, migration, and angiogenesis of endothelial progenitor cells, providing a protective effect against ischemic stroke [39]. The IL-17 signaling pathway contains the metzincin family, including matrix metalloproteinase-9 (MMP-9) and MMP-3. MMP-9 is involved in immune and inflammatory responses, as well as in disruption of the blood-brain barrier (BBB) and the promotion of leukocyte extravasation into the brain parenchyma [40]. Inflammation is currently considered a prime target for stroke therapies, and several preclinical studies have demonstrated the effectiveness of drugs targeting inflammatory factors, such as TNF, interleukin (IL)-6, and IL-10 [41]. Moreover, microglia-derived TNF-*α* mediates endothelial necroptosis and exacerbates BBB disruption after ischemic stroke [42].

RETRACTED

### 3.4. Uncovering the Key Antistroke Ingredients in AGNHW

Although AGNHW has shown a positive protective effect against stroke, the relevant MOA is unclear because the composition of the TCM formula is complex. To explore the material basis of AGNHW against stroke, we further narrowed the scope of the study of compounds in AGNHW to identify the key antistroke ingredients. Our statistical network model predicted that 128 compounds (adjusted *P*(*q*) < 0.01) in AGNHW with a high likelihood for stroke protection (Supplementary Table 5). Among them, 30 ingredients had known neuroprotective effects (Table 1) following a review of the available literature. For instance, sanguinarine exerts neuroprotective effects and anti-inflammatory effects following cerebral ischemia in rats [43], while acacetin has a protective effect against cerebral ischemia-reperfusion injury via the NLRP3 signaling pathway [44]. Interestingly, we found that 8 out of the 30 ingredients, including CA, SCU, chrysin, fisetin, gallic acid, imperatorin, morin, and palmatine, had not been proven to exert definite antistroke pharmacological effects after in-depth literature mining and deserve further investigation.

### 3.5. Evaluation of Drug-Like Properties and Pharmacological Validation of Potential Antistroke Ingredients In Vitro

We then evaluated the drug-like properties (Figure 5) of the eight candidate ingredients mentioned above. The proper range of the physicochemical properties was determined by the ADMETlab 2.0 [45]. By comprehensively considering the network-based predicted ranking, chemical structure, physicochemical properties, availability, and accessibility, these promising ingredients were selected for antistroke efficacy evaluation (Figure 5). Subsequently, the OGD/R injury model, a recognized in vitro model in ischemic stroke research, was applied for pharmacological validation [46, 47]. As shown in Figure 6, the OGD/R insult group showed significantly lowered PC12 cell viability (*P* < 0.01), while CA (6.25, 12.5, and 25 *μ*M), SCU (1, 2, and 4 *μ*M), chrisin (1, 2, and 4 *μ*M), fisetin (12 *μ*M), gallic acid (6.25 *μ*M), imperatorin (1, 2, and 4 *μ*M), and palmatine (3.125, 6.25, and 12.5 *μ*M) increased the viability of PC12 cells (^∗^*P* < 0.05, ^∗∗^*P* < 0.01, and ^∗∗∗^*P* < 0.001, respectively). In particular, the survival rates of PC12 cells treated with CA (6.25, 12.5, or 25 *μ*M) and SCU (1, 2, or 4 *μ*M) increased after the toxicity test (Supplementary Table 6), indicating their excellent neuroprotective activity against stroke.

RETRACTED

### 3.6. Mechanism of Action of SCU and CA Acid on Stroke

Next, SCU and CA were selected to decipher their potential MOAs in stroke given that they showed better neuroprotective effects on PC12 cells and preferable drug-like properties. First, we extracted the DTIs of these two compounds as well as the protein-protein interactions (PPIs) from a comprehensive human protein interactome [48] and constructed a subnetwork of SCU and CA (Figure 7(a)). SCU, a flavonoid found in TCM, has been reported to have protective effects against neuronal injury [49]. However, the specific MOA of antistroke remains obscure. As depicted in Figure 7(a), SCU interacts with eight stroke targets (e.g., ALDH2) and 44 PPI partners (e.g., BDNF), providing a potential molecular mechanism. A growing body of evidence has demonstrated that ALDH2 overexpression conferred neuroprotection and led to a significant reduction in mitochondria-related apoptosis in both in vitro and in vivo cerebral ischemia models [50]. Moreover, a previous study revealed that stroke severity was negatively correlated with BDNF levels during the process of acute stroke [51].

Likewise, as the main constituent of the medium-chain triglyceride ketogenic diet, CA has various properties, such as anticonvulsant effects [52]. Figure 7(a) shows that CA acts on six stroke targets (e.g., TP53) and 42 PPI partners (e.g., PTGS2), suggesting its possible MOA. Indeed, it has been reported that the proallele of TP53 is related to vascular repair and has the ability to functionally recover from stroke [53]. In addition, a previous in vivo study demonstrated that knockdown of PTGS2 expression could repress the NF-*κ*B signaling pathway, which inhibits apoptosis and promotes proliferation, migration, and angiogenesis of endothelial progenitor cells, thus providing a protective effect in mice with ischemic stroke [39]. Intriguingly, we found that SCU and CA could collectively act on shared targets, such as CYP3A4 and CYP2C19, indicating their potential synergistic mechanisms.

RETRACTED

Next, we performed biological process (BP) and KEGG pathway analyses on all stroke genes in the subnetwork (Figure 7(a)).  Figure 7(b) shows three groups of biological processes covering 17 items, such as negative regulation of apoptotic signaling pathway in Group 1 and regulation of inflammatory response in Group 3. Emerging evidence has revealed that several other TCM formulas also exert antistroke potential by targeting these two biological processes. For instance, the MOA of the Xiaoyao San formula for treating ischemic stroke is related to antiapoptosis and activation of the PI3K/Akt pathway [54]. Moreover, QiShenYiQi prescription was found to be protective in a subacute stroke model partly via mediating the inflammatory response [55].

Meanwhile, Figure 7(c) displays the KEGG pathway annotations, most of which were associated with stroke. Taking the PPAR signaling pathway as an example, previous studies demonstrated that XQ-1H (a novel derivative of ginkgolide B) could alleviate ischemic stroke by balancing pro/anti-inflammatory microglia polarization via the PPAR*γ* pathway both in vivo and in vitro, providing an alternative medication for stroke [56]. HIF-1*α* also plays a key role in remote ischemic preconditioning against stroke, likely mediated by systemic modulation of the inflammatory response [57]. Taken together, these results indicate that SCU and CA may exert their effects via apoptotic signaling pathways and inflammatory responses. Therefore, we next determined whether these two compounds could ameliorate inflammatory injury and decrease apoptosis in the OGD/R cell model.

### 3.7. SCU/CA Ameliorated Inflammatory Injury Induced by OGD/R Insult

To determine whether SCU and CA are involved in inflammation, we analyzed the expression of inflammatory cytokines using the ELISA kits. As shown in Figure 8, the expression of IL-1*β* in the OGD/R group was notably upregulated compared to that in the control group. Compared to the OGD/R group, the CA (6.25, 12.5, or 25 *μ*M) and SCU (1, 2, or 4 *μ*M) groups showed significantly reduced expression of IL-1*β*. Moreover, the OGD/R damage group increased the generation of IL-6 and TNF-*α* (*P* < 0.01), while CA and SCU treatment significantly decreased the generation of IL-6 and TNF-*α*. These data demonstrated that CA and SCU could protect against OGD/R-induced neuronal cell injury via anti-inflammatory effects.

RETRACTED

### 3.8. SCU/CA Significantly Decreased Apoptosis following Ischemic Insult

TUNEL staining was performed to explore the inhibitory effect of CA/SCU on OGD/R-induced apoptosis in PC12 cells (Figure 9(a)). The number of apoptotic cells significantly declined after treatment with CA/SCU in PC12 cells under OGD/R conditions. Annexin V-FITC/PI staining followed by flow cytometry demonstrated that OGD/R significantly promoted the apoptosis of PC12 cells (Figure 9(b)), whereas CA and SCU significantly reversed the OGD/R-induced apoptosis in PC12 cells. These data revealed that CA and SCU treatment ameliorated OGD/R-induced cell injury and apoptosis.

### 3.9. Investigating the Synergistic Effect of SCU/CA

To further explore the relationship between SCU and CA, here, we applied a network-based approach for drug combination (SCU and CA) to check their synergistic effect. A key network-based methodology asserts that a drug combination tends to be therapeutically effective only if it has a specific relationship to the disease module (stroke), as displayed by the “Complementary Exposure” pattern in targets' modules of both drugs [58, 59] (**Figure**S1A). In other words, these two drugs (SCU and CA) can be considered therapeutically synergistic combinations if their drug module (drug targets) only overlap with the stroke module. However in this case, the two drug (SCU and CA) modules are separated in the human interactome [60]. The computational results (**Figure**S1B) suggested that they were captured by the “Single exposure” pattern in the human interactome network rather than the “Complementary Exposure” pattern, indicating that they had no synergistic effect.

## 4. Discussion

With the aging of society, popular unhealthy lifestyle and widespread exposure to cardiovascular risk factors, stroke morbidity in China is displaying explosive growth and is characterized by a younger trend [61]. Although several medications have shown therapeutic effects on stroke, concerns remain regarding the dependency on time, the risk of hemorrhagic transformation (HT), and high cost [62]. Therefore, the development of novel therapeutic strategies for stroke is urgently needed. Compared to single-target chemical drugs with substantial toxic side effects and poor therapeutic effects on complex diseases, TCM formulas, which comprise comprehensive medicinal compounds, have the advantages of multicomponent, multipathway, and multitarget synergies. AGNHW, a well-known formula in TCM, has been clinically used for the treatment of cerebral diseases (e.g., stroke) for centuries. Indeed, AGNHW has been shown to exert neuroprotective effects and protect rats from injury caused by cerebral ischemia-reperfusion [7]. However, its active ingredients and underlying mechanisms have not been comprehensively and systematically investigated.

RETRACTED

In this study, we developed a systems pharmacology-based framework to investigate the MOA of AGNHW against stroke and identify the key antistroke ingredients in AGNHW. First, we constructed a drug-target network by collecting formula ingredients and mapping the known and predicted targets. We next decoded the specific MOAs of AGNHW for stroke via data integration analysis, including network analysis and integrated pathway analysis. Our results suggest that ANGHW may participate in the regulation of several crucial molecular pathways related to stroke pathogenesis, including the IL-17, TNF, and PI3K/AKT signaling pathways. Cytokines of the IL-17 family are reported to play a crucial role in promoting the inflammatory response and inducing secondary injury poststroke [63]. A meta-analysis demonstrated that TNF-*α* is associated with the risk of stroke and represents a defensive factor for stroke in the Asian population [64]. The PI3K/AKT pathway is another key signaling pathway in TCM formulas to treat stroke, which is involved in reducing neuronal apoptosis and promoting cerebrovascular production after stroke [65].

To identify the key antistroke ingredients in AGNHW, we first conducted a network-based in silico prediction and highlighted 30 key ingredients. After in-depth literature mining, we found that 8 of the 30 identified ingredients had not been previously confirmed to exert definite antistroke pharmacological effects, including CA, SCU, chrysin, fisetin, gallic acid, imperatorin, morin, and palmatine. We further evaluated the drug-like properties and performed pharmacological validation of these potential antistroke ingredients, and SCU and CA were selected for further investigation. Finally, we determined the antistroke effects of SCU and CA using an in vitro model of PC12 cells. SCU and CA significantly inhibited inflammation and apoptosis from OGD/R-induced injury. However, network-based prediction for drug combination indicated that SCU and CA had no synergistic effect on stroke. Collectively, our results supported systems pharmacology-based prediction of the potential mechanism of SCU and CA in mediating antistroke effects.

## 5. Conclusion

In this study, we proposed a multiple systems pharmacology-based framework to identify the potential antistroke ingredients in AGNHW and explore the underlying mechanisms of action (MOA) of AGNHW against stroke from a holistic perspective. Our approach has several advantages. First, we clarified the potential MOAs of AGNHW against stroke. The integrated pathway analysis demonstrated that the effects of AGNHW against stroke were due to multiple active compounds that targeted the inflammatory response and apoptotic signaling pathways. Second, systems pharmacology helped to identify the main active compounds in AGNHW against stroke, and the effects and mechanism of two candidates (SCU and CA) were further validated in an ischemia-reperfusion injury model.

RETRACTED

Overall, this research proposes an integrative systems pharmacology approach to identify antistroke ingredients and demonstrate the underlying pharmacological MOA of AGNHW on stroke, which provides an alternative strategy to investigate novel TCM formulas on complex diseases.

## Figures and Tables

**Figure 1:** Systems pharmacology-based framework of An-Gong-Niu-Huang-Wan (AGNHW) for the treatment of stroke. Construction of drug-target network and pathway integration of AGNHW (a). In silico prediction of key antistroke ingredients in AGNHW (b and c). Network analysis and pharmacological validation of SCU and CA against stroke (d).

**Figure 2:** Overlap analysis of herbal ingredients and corresponding targets of AGNHW. Overlap analysis of herbal ingredients among the 11 herbs in AGNHW prescription (a). The corresponding numbers of ingredients for each herb were as follows: 55 (Bingpian, BP), 292 (Yujin, YJ), 8 (Shuiniujiao, SNJ), 37 (Niuhuang, NH), 101 (Shexiang, SX), 36 (Zhenzhu, ZZ), 155 (Huanglian, HL), 175 (Huangqin, HQ), 5 (Zhusha, ZS), 5 (Xionghuang, XH), and 255 (Zhizi, ZZI). Overlap analysis of the corresponding targets among the 11 herbs in AGNHW prescription (b). The thickness of connected lines between two herbs is proportional to the overlapped targets. The corresponding numbers of targets for each herb were as follows: 14 (Bingpian, BP), 31 (Yujin, YJ), 14 (Shuiniujiao, SNJ), 15 (Niuhuang, NH), 32 (Shexiang, SX), 8 (Zhenzhu, ZZ), 23 (Huanglian, HL), 32 (Huangqin, HQ), 8 (Zhusha, ZS), 6 (Xionghuang, XH), and 46 (Zhizi, ZZI).

**Figure 3:** Global drug-target network of An-Gong-Niu-Huang-Wan (AGNHW). Labels of the top ten compounds and targets with highest degrees are displayed. The label font size and node size are proportional to the degree. The compounds were classified into six chemical scaffold clusters, which are displayed in different colors.

**Figure 4:** Integrated stroke-related pathways of AGNHW and its functional therapeutic modules. The pathway integration was based on the targets of AGNHW and relative pathways in KEGG database.

RETRACTED

**Figure 5:** Drug structures and physicochemical properties of the eight key ingredients (CA, SCU, chrysin, fisetin, gallic acid, imperatorin, morin, and palmatine) in AGNHW.

**Figure 6:** Active ingredients of AGNHW improved cell viability after OGD/R-induced neurotoxicity. The viability of PC12 cells was tested by MTT assay after treatment with caprylic acid (CA) (a), scutellarein (SCU) (b), chrysin (c), fisetin (d), gallic acid (e), imperatorin (f), morin (g), and palmatine (h). Data from three independent experiments are expressed as the mean ± SD (*n* = 3). ^#^*P* < 0.05, ^##^*P* < 0.01 compared to the control group and ^∗^*P* < 0.05, ^∗∗^*P* < 0.01, ^∗∗∗^*P* < 0.001 compared to the OGD/R group.

**Figure 7:** Mechanism of action of SCU and CA on stroke. Drug-target and PPI networks of SCU and CA (a). Biological process analysis (b) and pathway enrichment analysis (c) of the stroke targets of SCU and CA.

**Figure 8:** SCU and CA alleviated OGD/R-induced neuroinflammation. Effects of SCU and CA on IL-1*β* (a), IL-6 (b), and TNF-*α* (c) levels in PC12 cells induced by OGD/R. These data are presented as the mean ± SD (*n* = 3). ^##^*P* < 0.01 vs. control group; ^∗^*P* < 0.05 and ^∗∗^*P* < 0.01 vs. OGD/R group.

**Figure 9:** SCU and CA inhibited OGD/R-induced apoptosis. Apoptotic cells were detected by TUNEL staining (a) (Scale bar = 100 *μ*m). PC12 cell apoptosis after treatment with various concentrations of SCU/CA was determined by flow cytometry (b). Data are expressed as the mean ± SD (*n* = 3). Each experiment was performed in triplicate. ^##^*P* < 0.01 vs. control group; ^∗^*P* < 0.05 and ^∗∗^*P* < 0.01 vs. OGD/R group.

**Table 1:** Key antistroke ingredients in AGNHW.

Compound	PubChem ID	Adj-*P* value	Herb	PMID
**Fisetin**	CID 5281614	3.70E-04	HL	33782648
**Gallic acid**	CID 370	4.44E-04	ZZI	31680647
Oleic acid	CID 445639	8.62E-04	YJ	6656890
Curcumin	CID 969516	1.63E-03	YJ	8145684
P-cymene	CID 7463	3.25E-03	BP, YJ, HL	5471840
Sanguinarine	CID 5154	4.11E-03	HL	245136
Eriodictyol	CID 440735	4.23E-03	HQ	8190663
**Palmatine**	CID 19009	6.86E-03	HL	7981182
**Morin**	CID 5281670	8.78E-06	SX	5446461
Baicalein	CID 5281605	2.63E-05	HQ	32418004
**Chrysin**	CID 5281607	6.83E-05	HQ	8114856
Naringenin	CID 932	8.69E-05	YJ	453191
**Imperatorin**	CID 10212	1.33E-04	ZZI	705395
Eugenol	CID 3314	1.33E-04	YJ, HQ, HL	7047211
Geraniol	CID 637566	1.81E-04	YJ	7022886
**Caprylic acid**	CID 379	1.81E-04	YJ	7592840
Myristic acid	CID 11005	2.43E-04	YJ, ZZI	17586
Acacetin	CID 5280442	1.82E-07	HQ	6352603
Genistein	CID 5280961	2.83E-07	ZZI	63799
**Scutellarein**	CID 5281697	7.07E-07	HQ	31444086
Caffeic acid	CID 689043	1.78E-06	YJ, ZZI	4407787
Heptadecanoic acid	CID 10465	2.26E-06	YJ	25411278
Arachidic acid	CID 10467	2.26E-06	YJ	971073
Docosanoic acid	CID 8215	2.26E-06	YJ	18026827
Carvacrol	CID 10364	4.88E-06	YJ, SX	33970850
Estragole	CID 8815	4.88E-06	SX	25465853
Linoleic acid	CID 5280450	1.81E-06	YJ	32862121
Apigenin	CID 5280443	3.93E-08	HQ, ZZI	30949912
Stearic acid	CID 5281	3.17E-09	YJ, ZZI	32663656
Quercetin	CID 5280343	1.80E-13	ZZI	34214302

Note: the compounds in bold refer to 8 ingredients without definite antistroke pharmacological effects after in-depth literature mining.

RETRACTED

## Data Availability

The data used to support the findings of this study are included within the article.

## Abbreviations

ADMET: Absorption, distribution, metabolism, excretion, and toxicity
AGNHW: An-Gong-Niu-Huang-Wan
bSDTNBI: Balanced substructure-drug-target network-based inference
CA: Caprylic acid
DMEM: Dulbecco's modified Eagle's medium
FBS: Fetal bovine serum
IL-6: Interleukin-6
IL-1*β*: Interleukin-1*β*
MOA: Mechanism of action
MTT: 3-(4 : 5-dimethylthiazol-2-yl)-2 : 5-diphenyltetrazolium bromide
NCEs: New chemical entities
OGD/R: Oxygen-glucose deprivation/reoxygenation
SCU: Scutellarein
TNF-*α*: Tumor necrosis factor-*α*
tPA: Tissue-type plasminogen activator.

## Supplementary Materials

Supplementary 1 Supplementary Table 1: 1,128 chemical ingredients of AGNHW were obtained from the data sources.

Supplementary 2 Supplementary Table 2: integration of 245 stroke disease genes.

Supplementary 3 Supplementary Table 3: drug-target interaction (DTI) network.

Supplementary 4 Supplementary Table 4: detailed pathway information of AGNHW.

Supplementary 5 Supplementary Table 5: the key antistroke ingredients with a high likelihood for stroke protection in AGNHW.

Supplementary 6 Supplementary Table 6: cell toxicity test of CA and SCU.

Supplementary 7 Supplementary Figure S1: network-based drug combinations for stroke therapy.

## References

[1] Xu H., Wang E., Chen F., Xiao J., Wang M. (2021). Neuroprotective phytochemicals in experimental ischemic stroke: mechanisms and potential clinical applications. *Oxidative Medicine and Cellular Longevity*.

[2] Virani S. S., Alonso A., Aparicio H. J. (2021). Heart Disease and Stroke Statistics-2021 Update: A Report From the American Heart Association. *Circulation*.

[3] Price C. J., Menon D. K., Peters A. M. (2004). Cerebral neutrophil recruitment, histology, and outcome in acute ischemic stroke: an imaging-based study. *Stroke*.

[4] Tseng Y. J., Hu R. F., Lee S. T. (2020). Risk factors associated with outcomes of recombinant tissue plasminogen activator therapy in patients with acute ischemic stroke. *International Journal of Environmental Research and Public Health*.

RETRACTED

[5] Wang G. H., Lan R., Zhen X. D., Zhang W., Xiang J., Cai D. F. (2014). An-Gong-Niu-Huang Wan protects against cerebral ischemia induced apoptosis in rats: up-regulation of Bcl-2 and down-regulation of Bax and caspase-3. *Journal of Ethnopharmacology*.

[6] Zhao L., Peng F., Guan B. (2015). Whether metal element-containing herbal formula Angong Niuhuang pill is safe for acute brain disorders?. *Biological Trace Element Research*.

[7] Tsoi B., Chen X., Gao C. (2019). Neuroprotective effects and hepatorenal toxicity of Angong Niuhuang wan against ischemia-reperfusion brain injury in rats. *Frontiers in Pharmacology*.

[8] Du X., Li C., Zhang S. (2022). Exploring the pharmacological mechanism of calculus bovis in cerebral ischaemic stroke using a network pharmacology approach. *Journal of Ethnopharmacology*.

[9] Tsoi B., Wang S., Gao C. (2019). Realgar and cinnabar are essential components contributing to neuroprotection of Angong Niuhuang Wan with no hepatorenal toxicity in transient ischemic brain injury. *Toxicol Appl Pharmacol*.

[10] Xue X., Qu X. J., Yang Y. (2010). Baicalin attenuates focal cerebral ischemic reperfusion injury through inhibition of nuclear factor kappaB p65 activation. *Biochemical and Biophysical Research Communications*.

[11] Zhang X., Zhang X., Wang C. (2012). Neuroprotection of early and short-time applying berberine in the acute phase of cerebral ischemia: up-regulated pAkt, pGSK and pCREB, down-regulated NF-*κ*B expression, ameliorated BBB permeability. *Brain Research*.

[12] Zhang W., Huai Y., Miao Z., Qian A., Wang Y. (2019). Systems pharmacology for investigation of the mechanisms of action of traditional Chinese medicine in drug discovery. *Frontiers in Pharmacology*.

[13] Fang J., Zhang P., Zhou Y. (2021). Endophenotype-based in silico network medicine discovery combined with insurance record data mining identifies sildenafil as a candidate drug for Alzheimer’s disease. *Nature Aging*.

[14] Fang J., Liu C., Wang Q., Lin P., Cheng F. (2018). *In silico* polypharmacology of natural products. *Briefings in Bioinformatics*.

[15] Li D., Cai C., Liao Y. (2021). Systems pharmacology approach uncovers the therapeutic mechanism of medicarpin against scopolamine-induced memory loss. *Phytomedicine*.

[16] Huang L., Xie D., Yu Y. (2018). TCMID 2.0: a comprehensive resource for TCM. *Nucleic Acids Research*.

[17] Zhang R. Z., Yu S. J., Bai H., Ning K. (2017). TCM-Mesh: the database and analytical system for network pharmacology analysis for TCM preparations. *Scientific Reports*.

[18] Kim S. K., Nam S., Jang H., Kim A., Lee J. J. (2015). TM-MC: a database of medicinal materials and chemical compounds in Northeast Asian traditional medicine. *BMC Complementary and Alternative Medicine*.

RETRACTED

[19] Ru J., Li P., Wang J. (2014). TCMSP: a database of systems pharmacology for drug discovery from herbal medicines. *Journal of Cheminformatics*.

[20] Liu Z., Cai C., Du J. (2020). TCMIO: a comprehensive database of traditional Chinese medicine on immuno-oncology. *Frontiers in Pharmacology*.

[21] O'Boyle N. M., Banck M., James C. A., Morley C., Vandermeersch T., Hutchison G. R. (2011). Open Babel: an open chemical toolbox. *Journal of Cheminformatics*.

[22] Fang J., Wu Z., Cai C., Wang Q., Tang Y., Cheng F. (2017). Quantitative and systems pharmacology. 1. In silico prediction of drug-target interactions of natural products enables new targeted cancer therapy. *Journal of Chemical Information and Modeling*.

[23] Wu Z., Lu W., Wu D. (2016). In silico prediction of chemical mechanism of action via an improved network- based inference method. *British Journal of Pharmacology*.

[24] Guo P., Cai C., Wu X. (2019). An insight into the molecular mechanism of berberine towards multiple cancer types through systems pharmacology. *Frontiers in Pharmacology*.

[25] Cai C., Wu Q., Hong H. (2021). *In silico* identification of natural products from Traditional Chinese Medicine for cancer immunotherapy. *Scientific Reports*.

[26] Tabakman R., Jiang H., Shahar I., Arien-Zakay H., Levine R. A., Lazarovici P. (2005). Neuroprotection by NGF in the PC12 in vitro OGD model: involvement of mitogen-activated protein kinases and gene expression. *Annals of the New York Academy of Sciences*.

[27] Vavilis T., Delivanoglou N., Aggelidou E. (2016). Oxygen-glucose deprivation (OGD) modulates the unfolded protein response (UPR) and inflicts autophagy in a PC12 hypoxia cell line model. *Cellular and Molecular Neurobiology*.

[28] Wu L., Wang Y., Li Z., Zhang B., Cheng Y., Fan X. (2014). Identifying roles of "Jun-Chen-Zuo-Shi" component herbs of QiShenYiQi formula in treating acute myocardial ischemia by network pharmacology. *Chinese Medicine*.

[29] Li Y., Ren M., Wang J. (2021). Progress in borneol intervention for ischemic stroke: a systematic review. *Frontiers in Pharmacology*.

[30] Yuan Y., Men W., Shan X. (2020). Baicalein exerts neuroprotective effect against ischaemic/reperfusion injury via alteration of NF-kB and LOX and AMPK/Nrf2 pathway. *Inflammopharmacology*.

[31] Tu F., Pang Q., Huang T., Zhao Y., Liu M., Chen X. (2017). Apigenin ameliorates post-stroke cognitive deficits in rats through histone acetylation-mediated neurochemical alterations. *Medical Science Monitor*.

[32] Gao N., Tang H., Gao L., Tu G., Luo H., Xia Y. (2020). CYP3A4 and CYP11A1 variants are risk factors for ischemic stroke: a case control study. *BMC Neurology*.

RETRACTED

[33] Sherman B. T., Huang D. W., Tan Q. (2007). DAVID Knowledgebase: a gene-centered database integrating heterogeneous gene annotation resources to facilitate high-throughput gene functional analysis. *BMC Bioinformatics*.

[34] Rashidian J., Iyirhiaro G. O., Park D. S. (2007). Cell cycle machinery and stroke. *Biochimica et Biophysica Acta*.

[35] Uzdensky A. B. (2019). Apoptosis regulation in the penumbra after ischemic stroke: expression of pro- and antiapoptotic proteins. *Apoptosis*.

[36] Jin R., Liu L., Zhang S., Nanda A., Li G. (2013). Role of inflammation and its mediators in acute ischemic stroke. *Journal of Cardiovascular Translational Research*.

[37] Zhou Z., Xu N., Matei N. (2021). Sodium butyrate attenuated neuronal apoptosis via GPR41/G*βγ*/PI3K/Akt pathway after MCAO in rats. *Journal of Cerebral Blood Flow and Metabolism*.

[38] Heras-Sandoval D., Perez-Rojas J. M., Hernandez-Damian J., Pedraza-Chaverri J. (2014). The role of PI3K/AKT/mTOR pathway in the modulation of autophagy and the clearance of protein aggregates in neurodegeneration. *Cellular Signalling*.

[39] Zhou Z., Lu C., Meng S. (2019). Silencing of PTGS2 exerts promoting effects on angiogenesis endothelial progenitor cells in mice with ischemic stroke via repression of the NF-*κ*B signaling pathway. *Journal of Cellular Physiology*.

[40] Vafadari B., Salamian A., Kaczmarek L. (2016). MMP-9 in translation: from molecule to brain physiology, pathology, and therapy. *Journal of Neurochemistry*.

[41] Lambertsen K. L., Finsen B., Clausen B. H. (2019). Post-stroke inflammation-target or tool for therapy?. *Acta Neuropathologica*.

[42] Chen A. Q., Fang Z., Chen X. L. (2019). Microglia-derived TNF-alpha mediates endothelial necroptosis aggravating blood brain-barrier disruption after ischemic stroke. *Cell Death & Disease*.

[43] Wang Q., Dai P., Bao H. (2017). Anti-inflammatory and neuroprotective effects of sanguinarine following cerebral ischemia in rats. *Experimental and Therapeutic Medicine*.

[44] Bu J., Shi S., Wang H. Q. (2019). Acacetin protects against cerebral ischemia-reperfusion injury via the NLRP3 signaling pathway. *Neural Regeneration Research*.

[45] Xiong G., Wu Z., Yi J. (2021). ADMETlab 2.0: an integrated online platform for accurate and comprehensive predictions of ADMET properties. *Nucleic Acids Research*.

[46] Xu S., Li Y., Chen J. P. (2020). Oxygen glucose deprivation/re-oxygenation-induced neuronal cell death is associated with Lnc-D63785 m6A methylation and miR-422a accumulation. *Cell Death & Disease*.

[47] Zhao L. P., Ji C., Lu P. H., Li C., Xu B., Gao H. (2013). Oxygen glucose deprivation (OGD)/re-oxygenation-induced in vitro neuronal cell death involves mitochondrial cyclophilin-D/P53 signaling axis. *Neurochemical Research*.

RETRACTED

[48] Fang J., Wu Q., Ye F. (2021). Network-based identification and experimental validation of drug candidates toward SARS-CoV-2 via targeting virus-host interactome. *Frontiers in Genetics*.

[49] Dong Y., Zhang X., Liu M. (2019). Hybrid molecules of scutellarein and tertramethylpyrazine's active metabolites for ischemic stroke. *Bioorganic & Medicinal Chemistry Letters*.

[50] Xia P., Zhang F., Yuan Y. (2020). ALDH 2 conferred neuroprotection on cerebral ischemic injury by alleviating mitochondria-related apoptosis through JNK/caspase-3 signing pathway. *International Journal of Biological Sciences*.

[51] Karantali E., Kazis D., Papavasileiou V. (2021). Serum BDNF levels in acute stroke: a systematic review and meta-analysis. *Medicina (Kaunas, Lithuania)*.

[52] Wlaz P., Socala K., Nieoczym D. (2012). Anticonvulsant profile of caprylic acid, a main constituent of the medium- chain triglyceride (MCT) ketogenic diet, in mice. *Neuropharmacology*.

[53] Rodriguez C., Sobrino T., Agulla J. (2017). Neovascularization and functional recovery after intracerebral hemorrhage is conditioned by the *Tp53 Arg72Pro* single-nucleotide polymorphism. *Cell Death and Differentiation*.

[54] Xu Y., Chen W., Chen Z., Huang M., Yang F., Zhang Y. (2021). Mechanism of action of Xiaoyao San in treatment of ischemic stroke is related to anti-apoptosis and activation of PI3K/Akt pathway. *Drug Design, Development and Therapy*.

[55] Wang Y., He S., Liu X. (2021). Galectin-3 mediated inflammatory response contributes to neurological recovery by QiShenYiQi in subacute stroke model. *Frontiers in Pharmacology*.

[56] Liu R., Diao J., He S. (2018). XQ-1H protects against ischemic stroke by regulating microglia polarization through PPAR*γ* pathway in mice. *International Immunopharmacology*.

[57] Yang J., Liu C., Du X. (2018). Hypoxia inducible factor 1*α* plays a key role in remote ischemic preconditioning against stroke by modulating inflammatory responses in rats. *Journal of the American Heart Association*.

[58] Fang J., Pieper A. A., Nussinov R. (2020). Harnessing endophenotypes and network medicine for Alzheimer's drug repurposing. *Medicinal Research Reviews*.

[59] Cheng F., Kovacs I. A., Barabasi A. L. (2019). Network-based prediction of drug combinations. *Nature Communications*.

[60] Zhou Y., Hou Y., Shen J., Huang Y., Martin W., Cheng F. (2020). Network-based drug repurposing for novel coronavirus 2019-nCoV/SARS-CoV-2. *Cell Discovery*.

[61] Sacco R. L., Kasner S. E., Broderick J. P. (2013). An updated definition of stroke for the 21st century: a statement for healthcare professionals from the American Heart Association/American Stroke Association. *Stroke*.

RETRACTED

[62] Meschia J. F., Brott T. (2018). Ischaemic stroke. *European Journal of Neurology*.

[63] Waisman A., Hauptmann J., Regen T. (2015). The role of IL-17 in CNS diseases. *Acta Neuropathologica*.

[64] Gu L., Wu G., Yan Y. (2013). The role of *TNF- α* 308G > a polymorphism in the risk for ischemic stroke. *The American Journal of the Medical Sciences*.

[65] Zheng T., Shi Y., Zhang J. (2019). MiR-130a exerts neuroprotective effects against ischemic stroke through PTEN/PI3K/AKT pathway. *Biomedicine & Pharmacotherapy*.

